# The baseline characteristics and interim analyses of the high-risk sentinel cohort of the Vietnam Initiative on Zoonotic InfectiONS (VIZIONS)

**DOI:** 10.1038/srep17965

**Published:** 2015-12-10

**Authors:** Juan J. Carrique-Mas, Ngo T. Tue, Juliet E. Bryant, Karen Saylors, Nguyen V. Cuong, Ngo T. Hoa, Nguyen N. An, Vo B. Hien, Pham V. Lao, Nguyen C. Tu, Nguyen K. Chuyen, Nguyen T.K. Chuc, Dinh V. Tan, Hoang Van V. Duong, Tran K. Toan, Nguyen T.Y. Chi, James Campbell, Maia A. Rabaa, Behzad Nadjm, Mark Woolhouse, Heiman Wertheim, Guy Thwaites, Stephen Baker

**Affiliations:** 1 Hospital for Tropical Diseases, Wellcome Trust Major Overseas Programme, Oxford University Clinical Research Unit, Ho Chi Minh City, Vietnam; 2 Centre for Tropical Medicine, Nuffield Department of Clinical Medicine, Oxford University, Oxford OX3 7BN, United Kingdom; 3 National Hospital for Tropical Diseases, Wellcome Trust Major Overseas Programme, Oxford University Clinical Research Unit, Ha Noi, Vietnam; 4 Global Viral, San Francisco, CA 94104 USA; 5 Preventive Medicine Centre Dong Thap Province, Cao Lanh, Vietnam; 6 Sub-Department of Animal Health Dong Thap Province, Cao Lanh, Vietnam; 7 Preventive Medicine Centre Dak Lak Province, Buon Ma Thuot, Vietnam; 8 Regional Animal Health Laboratory 5, Buon Ma Thuot, Vietnam; 9 Sub-Department of Animal Health Dak Lak Province, Buon Ma Thuot, Vietnam; 10 Hanoi Medical University, Ha Noi, Vietnam; 11 Ba Vi District Health Centre, Ha Noi, Vietnam; 12 Ba Vi District Veterinary Station, Ha Noi, Vietnam; 13 Centre for Immunity, Infection and Evolution, University of Edinburgh, Edinburgh EH9 3FL, United Kingdom; 14 Department of Medical Microbiology, Radboud University Medical Cente, Nijmegen 6500 HB, the Netherlands; 15 London School of Hygiene and Tropical Medicine, London WC1E 7HT, United Kingdom

## Abstract

The Vietnam Initiative for Zoonotic Infections (VIZIONS) includes community-based ‘high-risk sentinel cohort’ (HRSC) studies investigating individuals at risk of zoonotic infection due to occupational or residential exposure to animals. A total of 852 HRSC members were recruited between March 2013 and August 2014 from three provinces (Ha Noi, Dak Lak, and Dong Thap). The most numerous group (72.8%) corresponded to individuals living on farms, followed by slaughterers (16.3%) and animal health workers (8.5%). Nasal/pharyngeal and rectal swabs were collected from HRSC members at recruitment and after notifying illness. Exposure to exotic animals (including wild pigs, porcupine, monkey, civet, bamboo rat and bat) was highest for the Dak Lak cohort (53.7%), followed by Ha Noi (13.7%) and Dong Thap (4.0%). A total of 26.8% of individuals reported consumption of raw blood over the previous year; 33.6% slaughterers reported no use of protective equipment at work. Over 686 person-years of observation, 213 episodes of suspect infectious disease were notified, equivalent of 0.35 reports per person-year. Responsive samples were collected from animals in the farm cohort. There was noticeable time and space clustering of disease episodes suggesting that the VIZIONS set up is also suitable for the formal epidemiological investigation of disease outbreaks.

Southeast Asia is considered a ‘hotspot’ for emerging infectious diseases. Over recent years this region (including southeast China) has witnessed the emergence of major outbreaks of severe zoonotic disease such as SARS, nipah virus and avian influenza^1^,^2^. The region has a higher than average proportion of mortality due to communicable diseases including many zoonoses, antimicrobial-resistant pathogens and vector-borne diseases^3^ and remains an epicentre of highly pathogenic avian influenza (HPAI)^4^. The reasons for this high incidence of emerging zoonoses in southeast Asia are complex, and likely to include multiple demographic, geographical, climatic, economic and cultural factors as well as agricultural practices that create an environment conducive to the emergence and propagation of zoonotic diseases^5^.

VIZIONS (Vietnam Initiative on Zoonotic InfectIONS) is a multidisciplinary project aiming to understand the emergence of zoonotic viral pathogens in human populations^6^. VIZIONS is performing in-depth comparisons of viromes on both sides of the species barrier (i.e. humans and animals) with concurrent investigation of the behavioural and demographic factors driving pathogen transmission and disease emergence. VIZIONS has two distinct components, one hospital- and one community-based. The hospital-based component aims to identify pathogens that have already crossed the species barrier causing serious infections requiring hospitalization. The community component, termed ‘a high-risk sentinel cohort’ (HRSC), focuses on individuals perceived to be at particularly high risk of infection with zoonotic pathogens because of their occupational or residential exposure^6^. These cohorts include people living on farms (including farms raising non-domestic or ‘exotic species’ – termed ‘exotic animal farms’), slaughterers (pigs and poultry), animal health workers, restaurant workers and rat traders.

Farmers represent the most common population subgroup, since 68% of the Vietnamese population is rural (GSO, 2013), and small-scale animal farming represents a common source of livelihood in rural settings. The HRSC studies primarily aim at detecting viruses involved in episodes of milder disease (i.e. not requiring hospitalization) by simultaneous co-sampling of humans and animals as close as possible to the date of onset of disease and characterize the major risks associated with exposure to animals and consumption of animal food. Sampling in the HSRC and hospital components overlap in space and time to ensure that pathogens discovered in one study population can be investigated in the other.

Recruitment for the VIZIONS HRSC was initiated in March 2013, and by September 2014 HRSC studies were established in three provinces of Vietnam (Dong Thap, Ha Noi and Dak Lak), all with differing human and geographical landscapes (the Mekong Delta, the Red River Delta, the Central Highlands, respectively). The aims of this report are: (a) To describe the methodologies used for recruitment of HRSC members and associated data collection; (b) to describe the demographic characteristics and high-risk exposures (i.e. contact with animals, slaughtering and consumption) among the HRSC members across the three provinces; and (c) to provide a current update report on the episodes of clinical disease reported.

## Results

### General characteristics of the high-risk cohort members

A total of 852 HRSC members were recruited between March 2013 and August 2014 from three provinces (271, 299 and 282 from Ha Noi, Dak Lak, and Dong Thap, respectively). The most numerous group corresponded to those resident on farms (72.8%), followed by slaughterers (16.3%) and animal health workers (8.5%). There were two categories of HRSC members represented in only one province each: restaurant workers of restaurants specialized in exotic animal meat (n = 15, Ha Noi) and rat traders (n = 5, Dong Thap). Overall, 48.7% of cohort members were female; the median age was 38 years (Table 1). Children aged less than 18 were only represented in the farm cohort, comprising 16.6% of this group (n = 103; 27, 35 and 41 in Ha Noi, Dak Lak and Dong Thap, respectively). Interviews for baseline questionnaire were conducted on 420 individuals (128, 162 and 130 from Ha Noi, Dak Lak, and Dong Thap, respectively) since only the head of the household was interviewed on farms.

### Exposure to live animals in farms or households

The most common live animal exposures (defined as whether cohort members had kept at home or worked in a farm with any animal species over the previous year) were to chickens (70.7%), followed by dogs (66.7%), pigs (56.7%), cats (37.4%), ducks (20.4%), wild pigs (16.1%), Muscovy ducks (16.1%) and cattle (12.8%) (Table 2). Overall exposure to exotic animals (including any of the following: wild pigs, porcupines, monkeys, civet cats, bamboo rats and bats) was highest in Dak Lak HRSC members (53.7%), followed by Ha Noi (13.7%) and Dong Thap (4.0%). Differences in animal exposures were also detected according to the occupation of the cohort member. Among farm cohort members, exposure to pigs and chickens was 87.6% and 70.6%, respectively, in contrast with 30.1% and 23.3% among animal health workers, and 27.5% and 20.2% among slaughterers. Exposure to civet cats and bamboo rats was restricted to Dak Lak HRSC members, whereas continued exposure to bats was reported only in the Dong Thap HRSC (one farm) (Table 2).

### Slaughtering/cooking and consumption of exotic animal meat

Data on slaughtering/cooking of exotic animal meat was available for 366 cohort members (data was not available from Ha Noi slaughterers, animal health workers and exotic animal restaurant workers). A total of 67 (18.3%) reported having slaughtered exotic animals or handled/cooked exotic animal meat and 121 (33.1%) reported the consumption of meat from exotic species at least once within the previous year. Overall, the most common types of exotic animals slaughtered/cooked were, in decreasing order: wild pigs (7.9% HRSC members), rats (6.8%), porcupines (2.5%) and civet cats (1.1%). The types of exotic meat consumed by responding HRSC members were (from most to least common): wild pigs (24.4%), porcupines (8.5%), rats (6.2%) and deer (4.5%). Both exotic animal cooking/slaughtering and consumption of exotic animal meat were most common within Dak Lak province (21.6% and 65.4% HRSC members, respectively), followed by Dong Thap (14.6% and 14.6%) and Ha Noi (8.0% and 10.0%). Farmers were the HRSC members mostly commonly practicing the slaughter/cooking of exotic animal meat (20.1%), followed by animal health workers (13.1%) and slaughterers (9.3%). Three out of five rat traders reported slaughtering rats over the previous year, the remaining two having only been involved in trapping and selling (Table 3). A larger proportion of males than females reported having slaughtered exotic animals (11.7% vs. 4.5%, respectively) (*p* = 0.023; Chi squared test). There were no statistical differences between the proportion of males and females reporting consumption of exotic animal meat (34.3% vs. 32.9%; *p* = 0.880; Chi squared test).

### Consumption of raw animal blood

The consumption of raw blood products is a common practice in Vietnam and we perceive this activity as a “risk” for the consumption of pathogens with zoonotic potential. Overall, 112/418 HRSC individuals (26.8%) reported the consumption of raw blood at least once within the previous year. The prevalence of consumption among HRSC members differed substantially by province, with Ha Noi having the highest proportion (55/114; 48.2%), followed by Dak Lak (47/162, 29.0%) and Dong Thap (5/128, 3.9%). Of the differing occupations represented in the cohorts, farmers most frequently reported raw blood consumption (33.1%), followed by slaughterers (18.7%) and animal health workers (17.9%). A total of 87/264 (33.0%) males consumed raw blood vs. 25/154 females (16.2%) (*χ*^2^ = 13.0; *p* < 0.001). The males aged 46–65 years had the highest reported frequency of consumption of raw blood (42/102, 41.2%) compared to all other groups (70/316, 22.1%) (*χ*^2^ = 13.2; p < 0.001).

The raw blood dishes (termed ‘tiet canh’ in Vietnamese) reportedly consumed by the HRSC included dishes made from pig blood (87 HRSC members), followed by duck (41), muscovy duck (13), rabbit (7) and goat (5) blood. Other types of tiet canh dishes such as those made from beef, chicken, porcupine, horse or wild boar blood, each dish was reported to have been consumed by only one or two individuals. Cohort members were also asked about their attitudes regarding the health consequences of consuming raw blood dishes. Of 112 raw blood consumers, 88 expressed an opinion, with 70 (79.6%) indicating a belief that this dish is unhealthy, and 43 (48.9%) attributed previous episodes of sickness to consumption of tiet canh. Of the 306 non-raw blood consumers, 59 expressed an opinion, with 100% (59/59) indicating that tiet canh dishes were likely to cause diarrhoea.

### Biting and injuries as a result of working with animals

A total of 53/420 (12.6%) HRSC members reported having been bitten to the point of bleeding by a mammal, reptile or scorpion within the last five years. A higher proportion of males reported biting episodes compared with females, although the difference was not significant (15.0% vs. 8.4%; *p* = 0.189). The species responsible for biting of HRSC members included dogs (25 HRSC members), pigs (9), cats (4), porcupines (4), rats (3), reptiles or scorpions (sting) (3), wild boar (1) and rabbit (1). The rat trader group was the HRSC group with the highest proportion of members reporting having been bitten (60%), followed by animal health workers (23.3%), farmers (14.3%) and slaughterers (4.3%). None of the restaurant workers reported to have been bitten by animals. A total of 35.5% HRSC members reported bleeding injuries (mainly due to the use of knives and needles) while working with or cooking animals over the previous year. Slaughterers reported the highest frequency of bleeding injuries (66.9%), followed by restaurant workers (21.4%), animal health workers (20.5%), rat traders (20%) and farmers (19.6%) (Table 4). All incidents involved cutting using a knife while slaughtering or cooking, except three individuals that reported skin abrasion while working with animals.

### Biosafety practices among slaughterers

Data were available for 117/139 (84.1%) professional slaughterers regarding biosafety procedures including the use of personal protective equipment (PPE). Shower facilities at work were available for 44 slaughterers (37.6%), but only 28 (24.4%) reported using these facilities after their working shift. Overall, a higher percentage of slaughterers from Ha Noi (54.2%) reported using shower facilities after work than those from Dak Lak (20.9%) and Dong Thap (3.3%). A total of 40 slaughterers (33.6%) reported that they do not use any PPE. Overall, the regular use of PPE was most common among slaughterers in Ha Noi (83.3%), followed by Dak Lak (80.6%) and Dong Thap (16.7%). The most commonly worn PPE reported by slaughterers included face masks (56.3% of slaughterers), followed by boots (42.9%), gloves (39.5%), and mob caps (3.4%).

### Episodes of disease

At the point of this analysis HRSC members had been followed up for a total of 685.7 person-years (0.804 years per person on average). The number of reported disease episodes was 213 (i.e. an incidence rate of 0.35 incidents per person-year) in 115 individuals. Seventy-seven of the episodes of disease were in females, and 136 were in males (incidence rate ratio (IRR) = 1.86 [0.46–16.15]). In comparison to children (age < 18 years) (baseline), individuals aged 19–50 years had increased frequency of reporting (IRR = 2.07 [1.34–3.32]), but this trend was not the same for individuals over 50 years (IRR = 1.43 [0.86–2.45]). No incidents had been reported in Dak Lak at the time of analysis over an observation period of 79.2 person-years. In contrast, a total of 179 and 34 incidents had been reported for a period of 357.4 and 248.7 person-years in Dong Thap and Ha Noi, respectively (IRR = 4.4 [3.0–6.6]).

In Dong Thap province, slaughterers had the highest incidence rate of reporting (2.2 per person-year), followed by animal health workers (0.63), rat traders (0.32) and farmers (0.25). Compared with farmers at baseline, the IRR among animal health workers and slaughterers were significantly higher (IRR = 2.54 [1.68−3.77] and IRR = 8.76 [6.60−11.63], respectively). In contrast, rat traders were similar in terms of risk to farmers (IRR = 1.27 [0.22−4.13]).

Among Ha Noi HRSC members the incidence rate for different cohort members ranged from none (restaurant workers) to animal health workers (0.23 per person-year), although there was no statistical difference in reporting between any of the different groups (data not shown). Notably, the distribution of disease reporting across the provinces was skewed, with many individuals reporting repeated episodes of disease whilst others reported none; whereas 71 HRSC members reported one episode, the number of individuals reporting 2, 3, 4, or more episodes of disease was 21, 11, 5, and 7, respectively. With 83 episodes reported by a total of 23 individuals, the Dong Thap slaughterer HRSC group had the highest number of multiple reporters. A graphical representation of person-time of HRSC members as well as the time points of reports of episodes of disease is shown in Fig. 1.

The most commonly reported symptoms among episodes of disease were respiratory (93.9%), including coughing, sneezing/runny nose, sore throat and dyspnoea, in decreasing order. Other disease episodes included: fever (90.5%), headache (63.2%), body aches (41.1%), and digestive disorders (11.3%), including diarrhoea and vomiting/nausea.

### Clustering of disease by commune and household

We identified some clustering of disease by commune and household. An example of case clustering was observed in Commune A in Dong Thap province, with 19 households and 70 HRSC members. In this commune, 26 cohort members reported a total of 39 incidents. In most cases these disease episodes were a combination of fever and respiratory disease, with 12 of the 26 first episodes reported by individuals occurring between June and July 2013 (Fig. 2 and Table 5).

### Human and animal samples

As part of longitudinal surveillance, respiratory, enteric and blood samples were obtained from HRSC members at recruitment (n = 852) and after each reported episode (n = 213) of a suspected infectious disease. A total of 3,320 animals belonging to 24 species were sampled from a total of 189 farms (mean = 17.6; SD = 2.1 per farm) as part of baseline sampling in the three provinces. In addition, 849 animals were sampled as a result of responsive sampling on farms (116 episodes of disease) (mean 7.3; SD = 1.4 per episode of disease reported).

## Discussion

Mid-way through the implementation of this HRSC study within the VIZONS initiative, the stated recruitment target of individuals with potentially high risk for exposure to zoonotic infections at high risk of animal contact has been reasonably met (852 vs. an initial target of 1,000). Data from the baseline questionnaires identified a number of potential factors and behaviours that may potentially increase the risk of zoonotic disease transmission, although we note that their prevalence is highly variable between provinces and occupation.

With this interim analysis, we report a total of 33.1% HRSC members that had consumed ‘exotic animal meat’ including meat from wild boars, porcupines, deer and rats within the previous year. This prevalence is not dissimilar from results of a previous survey carried out in four central districts in Ha Noi, which reported a prevalence of 22.6% of individuals eating exotic animals products^7^. In Vietnam and elsewhere in southeast Asia and China, high income rather than poverty is a major driver of the consumption of exotic animal meat^8^,^9^, and therefore, we predict that this trend is likely to increase in the foreseeable future^10^. The most commonly reported exotic animal meat types consumed included pangolins, deer, wild boar and porcupine. It is unclear from this study what fraction of overall ‘exotic animal’ consumption corresponds to farmed or hunted animals. Most consumption was reported from Dak Lak, a province in the Central Highlands, which is the home of the highest number of farms raising ‘exotic’ animal species, but also has some of the greatest biodiversity in the country. In contrast with northern Vietnam, where several exotic animal meat restaurants operate, it is thought that the majority of exotic animal meat consumed in the Central Highlands is consumed in private homes. Over recent years, the Vietnamese government has granted a considerable number of licenses to allow farming of exotic animal meat species with the hope of reducing demand on hunted exotic animals; however, whether this can achieve the desired aims is unclear^11^. In addition to their use as a food source, some exotic animals are raised for the harvesting of organs that are believed to have medicinal properties, such as the scales of pangolins and the stomach of porcupines^12^. The zoonotic risks due to contact with and consumption of exotic animal species are unclear, but in addition to the commonly known zoonotic pathogens affecting domesticated livestock in Vietnam^13^, it is likely to include a wider range of known and unknown bacterial, parasitic (i.e. cysticercosis, trematodal infections) and viral diseases. In addition, available veterinary knowledge that can provide relevant advice to farmers and consumers with relevant animal husbandry, disease diagnostic and inspection support is lacking.

The data presented here show the extent to which consumption of raw pig blood is common in northern and central parts of Vietnam. Pig blood pudding (‘tiet canh’) is, among other raw pig products, a known risk factor for *Streptococcus suis* infection, the most common cause of meningoencephalitis in the country^14^. A relevant finding is the fact that a high proportion of blood pudding consumers are aware of the potential disease risks that this may entail. This suggests that important cultural factors are likely to drive ‘tiet canh’ consumption and consumers regard that the benefits of this practice offset the potential risks.

A particularly striking finding is the lack of use of PPE among a third of slaughterers. There were considerable differences in PPE use by province, with slaughterers in Dong Thap reporting the lowest levels of PPE use (17%). We do not know to what extent this is related to the high rate of notification of disease among Dong Thap slaughterers, but episodes of disease were reported among a higher proportion of slaughterers not using PPE (data not shown). We are not currently aware of any studies that have been conducted examining risks and perceptions of zoonotic disease among slaughterers in Vietnam. It is striking to see this low level of protective equipment even in spite of the widespread concern of infection with diseases such as avian influenza among this occupational group^15^.

The results presented here suggest that the VIZIONS HRSC studies should provide ample opportunities for educational and training programmes aimed at increasing awareness on food safety as well as professional training for individuals participating in animal slaughter. The number of episodes of potential infectious disease reported to date (0.35 per person-year) fell considerably below the initial expectation of one episode per person per year. The data collected indicates that it is realistic to expect a total of ~900 episodes of disease over the duration of the project (3 years). Establishing effective disease notification systems for the VIZIONS HRSC studies requires effective engagement with local communities as well as effective co-ordination among a number of administrative authorities competent in both human and animal health. These requirements, along with the wide geographical distribution of the HRSC studies, are the most challenging operational components of VIZIONS. Notification of potentially infectious episodes of disease varies considerably depending on occupation and province. For example, the observed higher reporting rate of slaughterers in Dong Thap is likely to partly be the result of more active surveillance consisting of weekly telephone calls to the abattoir asking workers about their health, whereas other cohorts were contacted less frequently (monthly) during the initial phase of the study. In contrast, the absence of disease episode reporting in Dak Lak was likely due to saturation of capacity; initially, the field teams were heavily involved in carrying out baseline visits, and initial reported episodes by this cohort were not checked for their potential infectious nature. By the time of writing this report (March 2015), 128 episodes of disease had been reported in that province.

More generally, there are several additional limitations that may affect disease reporting and, thus, the results and inferences drawn from this study. Firstly, many cohort members are particularly averse to having blood drawn, especially when they are unwell. Secondly, some farmers are reluctant to notify since responsive sampling involves the collection of specimens from animals; there is a concern that any notifiable disease detected (i.e. HPAI, H5N1 or Porcine Respiratory and Reproductive Syndrome (PRRS) may lead to drastic official action such as total depopulation. In addition, we suspect that non-farmer cohorts are more likely to report disease since they share work place and therefore it is more difficult to conceal episodes of disease.

The observed cluster of disease in one commune, such as the one described in Commune A in Dong Thap province, suggests opportunities for formal outbreak investigations. Information about the potential links between some of the reported cases may help to better target our subsequent molecular epidemiological investigations. We have initiated contact with public health field epidemiology experts, which will hopefully assist with outbreak investigations in the near future. This may require an expansion of the definition of the population at risk beyond the recruited cohorts.

In summary, the initiation of the HRSC component of the VIZIONS project has been challenging, but these efforts are likely to produce a unique data set and biological resource. Samples and epidemiological data are being successfully collected as planned concurrently from humans and their animals during periods of health and illness. The project has already shown high prevalence of a range of consumption habits (i.e. consumption of raw blood pudding) and other exposures (i.e. absence of PPE and high frequency of bleeding injuries among slaughterers) likely to be associated with risk of transmission of zoonotic disease. The full achievement of VIZIONS HRSC objectives will depend on both on-going staff commitment and the maintenance of high levels of engagement with the communities under study.

## Methods

### Study population and recruitment process

In all three provinces farmers and their relatives, pig and poultry slaughterers, and animal health workers were recruited. These specific groups were targeted as these are common occupations in rural Vietnam. Exotic animal farmers (excluding cold blooded animals), rat traders and workers of exotic meat restaurants were enrolled wherever possible. Although these occupations are not a constant feature across the geography of Vietnam, they are considered to be at a high risk of exposure to zoonotic viruses. In all types of HRSC only adults were recruited, except on farms where up to four family members were recruited. The target was to recruit 1,000 individuals across the whole study (i.e. ~330 per province), to be followed for 3 years. This was expected to generate ~3,000 clinical events (1 event per person per year). Since farmers are the predominant population group in these provinces, it was decided that farmers (engaged both in raising domestic and exotic species) should correspond to approximately 2/3 of the study cohort. The composition of the remaining, non-farm cohort was decided in agreement with each province separately. Given the sensitive nature of the study, strict random selection of participants was not possible. Initially, the Sub-Department of Animal Health (SDAH) sent letters to a large number (~500 per district) of randomly selected poultry, pig and cattle farmers in each of the participating districts, based on the animal farm census, inviting them to attend an introductory information meeting. These meetings (one per district) were carried out to inform farmers of the aims and methodologies of the study. Those farmers that expressed an interest during the meeting were later contacted and were invited to attend, together with their relatives, to the local health centre where they consented to the study and baseline sampling was conducted. Over the first 3–4 months, all farm households were visited by a member of the study team (a doctor or a nurse) to enquire about their health and remind them of the objectives of the study, in order to establish a trust relationship between the study team and farm HRSC members. Non-farm cohort members were reminded by a monthly call to the abattoir, slaughter-point, veterinary station or restaurant by the project team. Slaughterers were selected from the most important pig abattoirs and poultry slaughter points in each of the participating locations. A number of restaurant workers, rat traders and animal health workers were the result of convenient sampling in each of the study provinces. These types of cohort members were also invited to participate in an information meeting prior to enrollment. Informed consent was obtained from all subjects prior to enrollment. All sampling and testing procedures were carried out in accordance with guidelines that had previously been reviewed and approved by the relevant institutional ethics committees for human and veterinary medicine. This includes the Ethics Board of Dong Thap Hospital and the review board of sub-Department of Animal Health (for work carried out in Dong Thap); the Ethics Board Hospital of Tropical Diseases and the review board of the sub-Department of Animal Health (for work carried out in Dong Thap province) and the Hanoi Medical University and the review board of the sub-Department of Animal Health in Ha Noi (for work carried out in Ha Noi). In addition, all methods were approved by the Oxford Tropical Research Ethics Committee (OxTREC) (No. 157-12) in the United Kingdom.

### Questionnaires and data capture

Three types of questionnaires (available as Supplementary Material) were designed to collect relevant exposure and disease data from HRSC members: (1) baseline questionnaires; (2) annual update questionnaires; and (3) disease episode questionnaires. Baseline questionnaires and annual update questionnaires were administered to all adult cohort members at recruitment and yearly thereafter, respectively. In the case of HRSC members living on farms, questionnaires were administered to the adult person primarily responsible for raising the animals. The baseline questionnaire includes the following sections: (a) basic demographic and socioeconomic data on HRSC members; (b) previous and current medical conditions; (c) exposure to exotic and domestic animals (including contacts in the household/farm, as well as hunting); (d) high risk food exposures (slaughtering, cooking and consuming exotic animal meat and consumption of uncooked/raw blood); and (e) occupational injuries and bites. Most questions on exposure related to the year prior to recruitment. Annual update questionnaires are comparable to the baseline questionnaire except that they record data on medical conditions and exposures during the previous year and additionally include sections dealing with specific behaviours that may increase the risk of transmission among farming families, slaughterers and animal health workers. Episode questionnaires are administered following a clinical disease episode, and include questions on food exposures over the previous month and changes in animal exposures since the administration of the previous questionnaire. We report here exposures reported in the baseline questionnaires.

### Episodes of disease

HRSC members were instructed to notify a contact person (a medical doctor or a nurse) belonging to the Preventive Medicine Centre (PMC) of the province in the event of an episode of ill health. The contact person would make a decision as to whether the reported illness could potentially be a communicable disease. In that case the contact person would arrange a visit to the sick participant’s household within 24–48 hours to conduct ‘responsive sampling’. If the episode involved someone living on a farm, the PMC authorities would immediately notify authorities from the sub-Department of Animal Health who would co-ordinate animal sampling on the farm.

### Human and animal sampling

Consenting HRSC members are sampled at recruitment (baseline sampling) as well as at the end of years one to three (update sampling) as well as following notification of an episode of illness (responsive sampling). Individuals are asked to provide the following samples: (1) rectal swab, (2) combined nasal and pharyngeal swab and (3) blood sample. For farm cohort members, up to 15 warm-blooded animals (i.e. birds and mammals) present are sampled on each visit. Given the high diversity of the composition of animal populations on farms, the decision as to which animals and how many are to be sampled is based on the relative species composition on each farm. A scoring system has been developed to help in the decision of which animals are to be sampled from each farm, with exotic and large animals having a higher score than small domestic livestock (See Supplementary Material). The types of sample collected from each animal include: rectal/cloacal swab (or faeces); nasal swab, blood and feathers (poultry). In the event of sick animals and/or mortalities at the time of a visit, such animals are sampled with priority. In addition (pigs and poultry) samples from abattoirs/slaughter points where HRSC members have been recruited and rats purchased from markets (Dong Thap) are to be collected over the three year duration of the study. Rat sampling involves collection of 45 randomly selected rats per province from 3 different markets (15 rats from each of 1 randomly selected trader per market) every 3 months. It is expected that this will result in a sample size of 540 rats over the 3 year period. Pig sampling and poultry is based on the abattoirs and slaughter points from where the participants have been recruited (1 or 2 of each per province). The sampling requirements for pigs in each province include 15 randomly selected pigs every 6 months (target 90 pigs over the three year period). For poultry the target is 15 poultry (chickens or ducks, depending on what is present on the date of the visit) to be randomly selected every 6 months (target 90 poultry over the three year period).

### Statistical methods

Comparisons of proportions were performed using Chi-square tests. All farm locations were geo-referenced and episodes of disease were plotted over time using Qgis version 2.2 software (www.qgis.com). Comparisons of incidence rates were calculated using the Epicalc package in R (www.r-project.org).

We are grateful to all participating cohort members, staff at RAHO 5, SDAH and PMC in Dak Lak, Dong Thap and Ba Vi, and Hanoi Medical University. A strategic award from Wellcome Trust of Great Britain funded this work (WT/093724). SB is a Sir Henry Dale Fellow, jointly funded by the Wellcome Trust and the Royal Society (100087/Z/12/Z).

## Additional Information

**How to cite this article**: Carrique-Mas, J. J. *et al*. The baseline characteristics and interim analyses of the high-risk sentinel cohort of the Vietnam Initiative on Zoonotic InfectiONS (VIZIONS). *Sci. Rep.* **5**, 17965; doi: 10.1038/srep17965 (2015).

## Figures and Tables

**Figure 1:** Graphical representation of person-time followed up for the HRSC members. Each horizontal line represents the person-time experience of one HRSC member. A black dot (∙) represents a reported episode of disease in one HRSC member. Colour code: dark blue: slaughterers; acqua: restaurant workers; pale blue: farmers; dark red: animal health workers; pink: rat traders.

**Figure 2:** Commune location of households (farm cohorts) with individuals reporting clinical disease for the first time during June and July of 2014, Dong Thap province, Vietnam. Yellow = not reporting disease, red = reporting disease. The circle highlights the location of Commune A in Dong Thap province. (Maps created using Qgis version 2.2 software).

**Table 1:** Occupation and province of origin of the HRSC members recruited in three provinces from March 2013 to August 2014.

Occupation	Province	No. cohort members	Percent (%)	Females (%)	Median age Years [IQR]
Slaughterer	Ha Noi	42	4.9%	78.6%	42.5 [34.2–46.7]
	Dak Lak	67	7.9%	49.3%	41.0 [31.5–46.0]
	Dong Thap	30	3.5%	26.7%	33.0 [27.2–47.0]
Animal health worker	Ha Noi	12	1.4%	41.7%	34.0 [29.2–41.0]
	Dak Lak	31	3.6%	32.3%	34.0 [30.5–47.0]
	Dong Thap	30	3.5%	6.7%	33.0 [30.0–48.2]
Farm cohort member	Ha Noi	202	23.7%	54.0%	40 [24–49.7]
	Dak Lak	201	23.6%	49.3%	38.0 [22.0–50.0]
	Dong Thap	217	25.5%	48.8%	39 [25.0–52.0]
Restaurant worker	Ha Noi	15	1.8%	60.0%	30.0 [21.5–46.5]
Rat trader	Dong Thap	5	0.6%	20.0%	38.0 [32.0–41.0]
All	All	852	100.0%	48.7%	38.0 [26.0–49.0]

**Table 2:** Exposure of HRSC (N = 852) members to live animals present on farms or, in case of non-farmers, in household environment.

Animal species	Farm cohort member			Animal health worker			Slaughterer			Restau-rant worker	Rat trader	All HRSC members
	Ha Noi (n = 202)	Dak Lak (n = 201)	Dong Thap (n = 217)	Ha Noi (n = 12)	Dak Lak (n = 31)	Dong Thap (n = 30)	Ha Noi (n = 42)	Dak Lak (n = 67)	Dong Thap (n = 30)	Ha Noi (n = 15)	Dong Thap (n = 5)	
Chicken	86.8	81.6	93.8	58.3	35.5	13.3	38.1	20.9	3.3	42.9		70.7
Dog	82.4	81.1	79.5	41.7	38.7	3.3	35.7	31.3	16.7	28.6	60.0	66.7
Pig	91.2	26.4	92.4	41.7	32.3	6.7	31.0	13.4	3.3	7.1		56.2
Cat	36.6	53.7	49.1	8.3	22.6	3.3	11.9	17.9	13.3			37.4
Duck	21.0	11.9	42.9	16.7	3.2	6.7	2.4	11.9				20.4
Wild pig	9.8	53.7	1.8					1.5		28.6		16.1
Muscovy		20.9	33.5			3.3						13.6
Cattle	37.6	10.9		8.3	9.7		2.4	9.0				12.8
Pigeon	8.3	23.9	2.2	8.3	6.5			1.5		21.4		9.0
Goose	5.4	11.9	5.4	16.7				3.0		21.4		6.3
Porcupine	5.9	18.4	0.4							7.1		6.0
Buffalo	11.2	2.0						7.5				3.7
Goat		10.9	1.8		3.2			3.0		7.1		3.5
Deer		14.9								7.1		3.6
Rabbit		5.5	2.2							14.3		2.1
Monkey		2.0	1.3									0.8
Turkey		1.5	0.4									0.5
Civet		2.0										0.5
Quail		2.0										0.5
Bamboo rat		1.8										0.4
Bat			1.3									0.3

Data are expressed as percent of individuals in each cohort (%) in descending order by number of HRSC members exposed to specific animal species. Empty cells indicate no exposure reported.

**Table 3:** The proportion of interviewed HSRC members reporting slaughtering or cooking of exotic animals or consuming exotic animal meat.

Exotic animal species		Farmer			Animal health worker		Slaughterer		Rat trader	
		Ha Noi (n = 60)	Dak Lak (n = 64)	Dong Thap (n = 65)	Dak Lak (n = 31)	Dong Thap (n = 30)	Dak Lak (n = 67)	Dong Thap (n = 30)	Dong Thap (n = 5)	All HRSC members
Slaughtering or cooking	Wild pig	5.0	29.7		12.9	3.3	0.0	3.2		7.9
	Rat			7.7		10.0	19.4		60.0	6.8
	Porcupine	3.3	10.9							2.5
	Civet cat		3.1		6.5					1.1
	Bamboo		0.0	1.5					20.0	0.6
	Squirrel		1.6							0.3
	Deer		0.0		3.2					0.3
	Jungle fowl		1.6							0.3
	Pangolin		1.6							0.3
	Any species	8.3	42.2	9.2	16.1	10.0	19.4	3.2	80.0	18.3
Consuming	Wild pig	5.0	73.4	1.5	64.5	3.3		46.7		24.4
	Porcupine	5.0	28.1		19.4	3.3		6.6		8.5
	Rat			7.7	3.2	13.3	13.3	0.0	60.0	6.2
	Deer		12.5		19.4			6.6		4.5
	Civet cat		9.4		12.9			3.2		3.1
	Bamboo		3.1	1.5	12.9			3.2	20.0	2.5
	Squirrel		3.1		6.5					1.1
	Jungle fowl		1.6		3.2			3.2		0.8
	Bat		1.6					0.0		0.3
	Any species	10.0	84.4	10.8	64.5	13.3	13.4	46.7	80.0	33.1

Data are expressed as percent of individuals in each cohort (%) (data from 366 completed questionnaires). Empty cells indicate no exposure reported.

**Table 4:** The number and proportion of HRSC (%) reporting being bitten by an animal to the point of bleeding or having had a bleeding injury when working with animals and its frequency over the previous 5 years (data from 366 completed questionnaires).

	Bitten	Other bleedinginjuries	No. of other bleeding injuries/year			
			1	2–3	4–12	>12
Farmer	27 (14.3)	37 (19.6)				
Ha Noi (n = 60)	5 (8.3)	12 (20)	2	5	5	
Dak Lak (n = 64)	14 (21.9)	20 (31.3)	9	8	3	
Dong Thap (n = 65)	8 (12.3)	5 (7.7)	1	2	2	
Animal health worker	17 (23.3)	15 (20.5)				
Ha Noi (n = 12)		1 (8.3)		1		
Dak Lak (n = 31)	8 (25.8)	10 (32.3)	4	5	1	
Dong Thap (n = 30)	9 (3)	4 (13.3)	2	2		
Slaughterer	6 (4.3)	93 (66.9)				
Ha Noi (n = 42)		18 (42.9)	1	3	12	2
Dak Lak (n = 67)	2 (3.0)	51 (76.1)	3	30	10	8
Dong Thap (n = 30)	4 (13.3)	24 (8)	2	16	3	3
Rat trader	3 (6)	1 (20)				
Dong Thap (n = 5)	3 (6)	1 (2)			1	
Restaurant worker		3 (21.4)				
Ha Noi (n = 15)		3 (21.4)		1	2	
	53 (12.6)	149 (35.5)	24	72	38	13

Empty cells indicate no bleeding injuries reported.

**Table 5:** Reporting of episodes of disease among cohort members in Commune A (only first report for each individual shown).

Household	No. household members	No. membersreporting disease	Onset (first report of each member)	Symptoms reported*
75–36	4	4	30/07/13, 11/05/14, 1/06/14 (2)	FRB, FRH, FDB, FRH
75–37	3	0	–	
75–38	4	3	20/06/13	FRB, FRH, FR
75–39	4	2	18/04/14	FDB, S
75–40	3	0	–	
75–41	4	2	06/12/13, 01/06/14	FR, FRBH
75–42	4	0	–	
75–43	4	3	20/06/13 (2); 30/09/13	FR, FR, FRB
75–44	3	0	–	
75–45	4	2	06/06/13, 01/06/14	FR, FRH
75–46	3	1	01/06/14	FRBH
75–47	4	1	06/06/13	FRB
75–48	4	1	10/07/13	FR
75–49	3	1	20/06/13	FRBH
75–50	4	1	10/07/13	FRH
75–51	4	2	20/06/13 (2)	FRBH, FRDBH
75–52	4	0		
75–53	4	3	30/07/13	FRB (2), FRBH
75–54	3	0	–	
Total	70	26		

*F = fever; R = respiratory signs; B = body ache; H = headache; D = digestive signs; S = skin disorders.
